# Bone marrow mesenchymal stem cells inhibit dendritic cells differentiation and maturation by microRNA-23b

**DOI:** 10.1042/BSR20160436

**Published:** 2017-04-20

**Authors:** Jingguo Wu, Chengbo Ji, Feifei Cao, Hongfen Lui, Bo Xia, Lanping Wang

**Affiliations:** 1 Department of Orthopedics, Affiliated Hospital of Taishan Medical University, Taian 271000, Shandong Province, China; 2 Department of Orthopedics, Taian City Centre Hospital, Taian, 271000, Shandong Province, China; 3 Department of Nursing, Taian City Centre Hospital Branch, Taian, 271000, Shandong Province, China

**Keywords:** bone marrow mesenchymal stem cells (BMSCs), dendritic cells (DCs), immune tolerance, miR-23b, maturation, NF-κB pathway

## Abstract

Research on regulation and its mechanism of bone marrow mesenchymal stem cells (BMSCs) on dendritic cells (DCs), which is the initiating factor in immune response has applicable clinical value. Although BMSCs have a significant regulatory effect on the maturation of DCs, its molecular mechanism is still unclear. BMSCs and DCs, were co-cultured by different concentration ratios. Flow cytometry was used to detect the expression of DC markers (CD83, CD11c). Quantitative reverse transcription PCR (qRT-PCR) was used to measure the expression of related genes in RNA level. Expression of the target proteins was detected with using Western blot assay. miRNA inhibitor and miRNA mimic were used to suppress and up-regulate the expression of the target gene. In this research, our results demonstrated that BMSCs notably inhibited maturation of DCs in the co-culture system of BMSCs and DCs and confirmed that this inhibition is due to overexpression of *miR-23b*. Furthermore, this research found that *miR-23b* overexpression inhibited the expression of p50/p65, thus blocked the activation of the NF-κB pathway. In conclusion, BMSCs affected the activation of NF-κB pathway through *miR-23b* overexpression resulting in inhibition of the maturation and differentiation of DCs.

## Introduction

Bone marrow mesenchymal stem cells (BMSCs) are multipotent non-haematopoietic adult stem cells, which are derived from the embryonic mesoderm. They can be highly self-renewable and have multidirectional differentiation potential. Because of the characteristics of BMSCs, including low immunogenicity [1], haematopoietic reconstitution [2], immunomodulation [3] and so on, they are ideal seed cells for transplantation, especially in bone tissue engineering. BMSCs have specific immunological properties, which can inhibit the proliferation and function of lymphocytes and then suppress immunoreaction and induce immune tolerance [4]. BMSCs were co-cultured with CD19^+^ B cells and found that the proliferation of B cells was obviously inhibited [5]. Studies have confirmed that BMSCs could secrete a large amount of CXCL12 that was the chemokine of CD8^+^ memory cells homing [6]. Obviously, BMSCs immune regulation is characterized by multiple pathways and mechanisms and mainly through two ways of secretion of immune regulatory factors and direct contact between cells. Although the immune regulation of BMSCs is a new hotspot in the field of transplantation, its specific mechanism is still unclear.

Dendritic cells (DCs) are a kind of antigen-presenting cells which have important function *in* *vivo* [7]. Since DCs are the initial factors of the immune response to activate naive T cells [8], they have an indispensable role in the immune response. However, DCs play a dual role in the regulation of immune responses [9]. On the one hand, DCs can induce graft rejection. On the other hand, DCs are also able to regulate T-cell responses, resulting in immune tolerance which has great significance for the treatment of autoimmune diseases, transplant rejection and allergic diseases. The maturity state of DCs is closely related to the type and extent of immune response induced by it [10]. Mature DCs usually induce immune activation. Due to the lack of second signal expression on the immature DCs (iDCs) surface, it can lead to apoptosis of antigen-specific T cells, which can induce the antigen-specific tolerance. From the mechanism of DCs induced immune tolerance, the way to increase the tolerance of DCs is to inhibit their maturation. In addition to some drugs and cytokines, BMSCs have also been shown to affect DCs differentiation and maturation, thus processing its immune regulatory function [11].

Currently, more and more studies have identified that miRNAs play an important regulating role in the maturation and differentiation of immune cells and immune response [12]. *miR-148*, *miR-142*, *miR-146a* and *miR-29a* have been confirmed to be related to DCs maturation and function [13]. In addition, studies have indicated that fibroblasts could promote DCs maturation; while the expression of miR-23b in fibroblasts was markedly lower than in BMSCs [14]. However, BMSCs with regulatory role for DCs maturation had a high expression of *miR-23b* [15]. It is believed that the expression of *miR-23b* is associated with DCs maturation.

Although BMSCs have a significant regulatory effect on the maturation of DCs, its molecular mechanism is still unclear. Combined with previous research results, we confirmed the important role of *miR-23b* in this regulation mechanism and investigated the underlying molecular mechanisms of *miR-23b*.

## Materials and methods

### Cell culture

#### BMSCs culture

The cells were isolated and cultured as recently described [16]. BALB/C mice bone marrow was collected and anticoagulated with heparin, and Ficoll discontinuous density gradient centrifugation (2000 rpm, 20 min) was used to harvest mononuclear cells from bone marrow. The cells were washed with PBS (HyClone) and then were suspended in low glucose DMEM (Gibco) medium containing 10% FBS (Gibco) and 1% penicillin-streptomycin (P/S, HyClone). The cell suspension was inoculated into 100-ml cell culture flask (Corning) with 1 × 10^6^ cells/ml density and cultured (37°C, 5% CO_2_). After 4–6 days of culture, the culture medium was replaced to remove the non-adherent cells. The adherent cells were sequentially cultured and we changed the growth medium every 3 days. When the cellular fusion rate was 80–90%, the cells were digested with trypsin and carried out subculture. Animal experiments were carried out strictly in accordance with the guidelines of the experimental animal management of the Affiliated Hospital of Taishan Medical University.

#### iDCs culture

As previously described [17], C57BL/6 mice peripheral blood was collected and anticoagulated with heparin,༌and Ficoll discontinuous density gradient centrifugation (2000 rpm, 20 min) was used to harvest mononuclear cells from bone marrow. The cells were washed with PBS (HyClone) and then were resuspended in RPMI-1640 (Gibco) medium containing 10% FBS (Gibco) and 1% P/S (HyClone). The cell suspension was inoculated into six-well plates (Corning) with 6 × 10^6^ cells/ml concentration and cultured (37°C, 5% CO_2_). After 2 h of incubation, non-adherent cells were discarded and RPMI-1640 culture medium was used to wash the remaining adherent cells. We cultured adherent cells with medium containing recombinant rat GM-CSF (50 ng/ml) (PeproTech) and recombinant rat IL-4 (50 ng/ml) (Invitrogen) at 37°C, 5% CO_2_. On the third and the fifth day, 1 ml fresh medium was added to each cell culture system and collected the suspended cells at the seventh day.

#### Lymphocytes culture

Lymphocytes were isolated as in a recent study [18]. Briefly, the peripheral blood mononuclear cells were cultured for 2 h with RPMI-1640 medium (HyClone) containing 10% FBS (Gibco) and 1% P/S (Hyclone) and the suspended cells were lymphocytes.

### Transwell co-culture of DCs and BMSCs

MSCs and DCs were placed in the upper and lower layers of the six-well Transwell plate, respectively, in different proportions (1:100, 1:50, 1:25, 1:10) for 48 h. Each well contained 5 × 10^5^ DCs in the Transwell plate. The culture medium used in these co-culture systems was composed of RPMI-1640 medium, FBS (10%), recombinant rat IL-4 (50 ng/ml), recombinant rat GM-CSF (50 ng/ml), LPS (200 ng/ml, Sigma) and TNF-α (10 ng/ml, Sigma). LPS and TNF-α were used to stimulate iDCs maturation.

### Flow cytometry analysis

As previously described [16,19], cells in the co-culture system of DCs and BMSCs were digested with 0.25% trypsin (HyClone) and collected and then washed twice with PBS. After centrifugation, the supernatant was discarded and the cells were resuspended in the EP tubes, 100 μl, 2 × 10^5^ cells per tube. Added 1 μl of anti-CD83-PE antibody (BD PharMingen), anti-CD11c-FITC antibody (BD PharMingen) and isotype control antibody (BD PharMingen) to the EP tube respectively. After incubation for 30 min in the dark at 4°C, the cells were washed twice with PBS and then resuspended in 0.2 ml PBS. Flow cytometry (Thermo Scientific) was used to detect DCs phenotype changes, and the experimental results were analysed using Guava Incyte (GuavaSoft V2.7, Millipore) analysis software.

### Quantitative real-time PCR

Quantitative reverse transcription PCR (qRT-PCR) was performed as previously described [20]. Cells were harvested, total RNA was extracted with TRIzol kit (Invitrogen), and the concentration was determined under the guidance of the manufacturer. cDNA was synthesized by reverse transcription with the same amount of RNA in each experimental group. Expressions of related genes were detected by SYBR fluorescent staining PCR with DyNAmo HS SYBR Green qPCR Kit (Thermo Scientific). The relative expression of the gene in the cells was calculated with 2^–།ΔΔ*C*^_t_ and β-actin as internal reference. The amplification process was 94°C for 2 min, 94°C for 20 s and 60°C for 57 s, a total of 40 cycles. Detection of target gene amplification level was by ABI 7500 PCR Real-Time System (Applied Biosystems). The special primers were designed and synthesized by Sangon Biotech.

### Transfection of cells with *miR-23b* inhibitor/mimics

Cells were grown in 12-well plates at 2.5 × 10^5^ cells per well and the fusion rate was approximately 70–80%. *miR-23b* inhibitor/mimics (2.5 μl, 8 × 10^4^ nM) and Lipofectamine TM 2000 Reagent (2.5 μl) were sequentially added to 100 μl serum-free culture medium and let it stand for 5 min. The mixed solution was added into the cells and expanded to 1 ml with serum- and antibiotic-free medium. After 4 h of culture, the culture medium was discarded. The transfected cells were used in the following experiments. All of the inhibitors, mimics and liposomes in the present study were purchased from Ribobio, Guangzhou.

### Mixed lymphocyte reaction

DCs lost their proliferative capacity by mitomycin C (25 μg/ml) pretreatment for 30 min. The co-culture systems of DCs and BMSCs that were pretreated with *miR-23b* inhibitor/miRNC were established and then co-cultured with lymphocytes (1:10) for 72 h. After culture, MTT was added to the cells, and then we removed the cell culture supernatant and supplemented the cells with DMSO after 4 h. The proliferation of lymphocytes was detected by microplate reader (Bio–Rad Laboratories) at 490 nm.

### Western blotting

Western blotting was performed as previously described [21]. Cells’ total protein was extracted with lysis buffer (Invitrogen), and the target proteins were separated from total protein by SDS/PAGE. The target proteins on gel were transferred to the PVDF membrane (Millipore). BSA (Gibco) sealed up PVDF membrane for 2 h, proteins were marked by primary antibodies anti-p65 antibody (1:1000, Abcam) or anti-p50 antibody (1:10000, Abcam) or anti-β-actin antibody (1:2000, Abcam) and anti-rabbit HRP secondary antibodies (1:1000, Abcam). PVDF membrane was washed with PBS and we observed the chemiluminescence with ECL Plus Western Blotting Substrate (Thermo Fisher). The film that was placed on the PVDF membrane was exposed and developed.

### Statistical analysis

The data were derived from three or more independent experiments. Statistical analysis was performed by GraphPad Prism with one-way ANOVA and Student’s *t*-test (*P*<0.05).

## Results

### BMSCs inhibited maturation of DCs

The results showed that the expressions of CD83, CD11c, CD80, CD86, HLA-DR, MHC-II and OX62 were significantly decreased when the co-culture ratio of BMSCs and PBMCs was 1:50 (Figure 1A, B); moreover, the expression of IL-12 was significantly decreased and IL-10 was significantly increased. And the inhibition of DCs maturation was increasing as the proportion of BMSCs in co-culture system was increasing (Figure 1C).

**Figure 1:** BMSCs inhibited maturation of DCs BALB/C mice-derived BMSCs and C57BL/6 mice-derived PBMCs (with the tendency to differentiate into DCs) were co-cultured *in vitro* with 1:100, 1:50, 1:25 and 1:10 respectively. (**A**) After 48 h of culture, the expressions of DCs maturation markers CD83 and CD11c were analysed by flow cytometry. (**B**) The expressions of the cell surface markers were significantly decreased when the co-culture ratio was 1:50 or 1:25 or 1:10. (**C**) The expression of IL-12 was significantly decreased and IL-10 was significantly increased when the co-culture ratio of BMSCs and PBMCs was 1:50; *P<0.05.

### *miR-23b* was highly expressed in BMSCs

We compared the expression of *miR-23b* in BMSCs and it was significantly higher than that in osteo-differentiated mesenchymal stem cells (MSCs) and fibroblasts (Figure 2A). When BMSCs were transfected with *miR-23b* inhibitor, *miR-23b* expression was significantly decreased indicating that its expression was effectively inhibited (Figure 2B).

**Figure 2:** *miR-23b* was highly expressed in BMSCs (**A**) The expression of *miR-23b* in BMSCs was the largest and significantly different from that in osteo-differentiated MSCs and fibroblasts. (**B**) BMSCs were transfected with *miR-23b* inhibitor, followed by a significant decrease in *miR-23b* expression compared with control groups; *P<0.05.

### Effects of *miR-23b* expression on DCs maturation and lymphocytes proliferation

In the present study, we further explored the maturity of DCs under different culture conditions. The obtained results of detecting DCs mature markers revealed that the co-cultured BMSCs with DCs (with 1:25 ratio) has obvious inhibitory effect on the maturation of DCs compared with the cultured DCs alone; however, in the co-culture of DCs and BMSCs that transfected with *miR-23b* inhibitor, the maturation of DCs was not significantly inhibited (Figure 3A,C,D). The lymphocytes were cultured in different culture systems of DCs in order to investigate the effect of *miR-23b* expression on lymphocytes proliferation. Lymphocytes had a high proliferation rate when they were co-cultured with DCs. In co-culture systems, BMSCs significantly inhibited the proliferation of lymphocytes. Lymphocytes proliferation was not significantly inhibited when co-cultured with BMSCs pretreated with *miR-23b* inhibitor (Figure 3B).

**Figure 3:** Effects of *miR-23b* expression on DCs maturation and lymphocytes proliferation (**A,C,D**) BMSCs were pretreated with *miR-23b* inhibitor and then BMSCs and DCs were co-cultured with 1:25 ratio, DCs maturation was significantly promoted. (**B**) DCs with different treatment conditions were co-cultured with lymphocytes (with 1:10 ratio) for 72 h. When DCs were co-cultured with BMSCs and the expression of *miR-23b* was inhibited, the lymphocytes proliferation rate was significantly higher; *P<0.05.

### Expression of *miR-23b*, p50 and p65 under different culture conditions

The expression of *miR-23b* was significantly increased in the co-culture condition of DCs and BMSCs compared with the cultured DCs alone; when BMSCs were transfected with *miR-23b* inhibitor, the expression of *miR-23b* in co-culture system also decreased obviously (Figure 4A). The co-culture of DCs and BMSCs with *miR-23b* inhibitor significantly relieved the inhibitory effect of BMSCs on the expression of p50 and p65, and the expressions of p50 and p65 were significantly increased at the level of gene (Figure 4B, C) and protein (Figure 4D). The expressions of p50 and p65 were significantly decreased with *miR-23b* overexpression in the co-culture system in protein level (Figure 4D).

**Figure 4:** Expression of *miR-23b*, p50 and p65 under different culture conditions Pretreatment with *miR-23b* inhibitor for BMSCs (**A**) reversed the high expression of *miR-23b* induced by co-culture of BMSCs and DCs and the expression of *miR-23b* was significantly decreased; meanwhile, compared with the control group the expression of (**B**) p50 and (**C**) p65 increased remarkably with the inhibition of *miR-23b* expression. (**D**) In protein level, the expressions of p50 and p65 were notably increased when the expression of *miR-23b* was inhibited; *P<0.05.

### The relationship between the expression of *miR-23b* and p50/p65 in DCs

The results showed that *miR-23b* overexpression inhibited both the expression of p50 and p65, and the expressions of p50 and p65 were significantly increased after *miR-23b* expression was inhibited (Figure 5A, B). Obviously, the relationship between the expression of *miR-23b* and p50/p65 was negative correlation.

**Figure 5:** The relationship between the expression of *miR-23b* and p50/p65 in DCs (**A**) In both the gene and (**B**) protein levels, *miR-23b* overexpression inhibited the expression of p50/p65, while down-regulated *miR-23b* expression promoted the expression of p50/p65; *P<0.05.

## Discussion

Since DCs were first reported in 1973, their related researches have been concerned by the immunology. T-cell response is a key point in the host immune response or tolerance for antigen [22], and DCs are the only antigen-presenting cells that can activate the naive T cells [23]. Therefore, DCs play an important role in the process of inducing T-cell activation or tolerance. Mature DCs can effectively activate T cells and are considered to be important mediators to allogeneic transplantation rejection [24]. iDCs are responsible for the induction of tolerance to specific antigen T cells in the immune system [25]. Some studies have found that iDCs can promote the survival of cardiac allograft without the use of immunosuppressant [26]. iDCs inhibited the occurrence of acute graft compared with host disease (GVHD) after allogeneic bone marrow transplantation [27] and it also can reduce the relapse of leukaemia [28]. The immune regulation of BMSCs is a new hotspot in the field of transplantation, and its inhibition on T lymphocytes proliferation has been generally recognized. Research on regulation and its mechanism of BMSCs on DCs that are the initiating factors in immune response has the important research significance in the present study. In this research, our results demonstrated that BMSCs notably inhibited maturation of DCs in the co-culture system of BMSCs and DCs. This conclusion was consistent with the results of Ramasamy et al. [11]. This suggested that BMSCs may play the role of immune regulation by inhibiting the maturation of DCs.

Studies have indicated that fibroblasts that have relatively low expression of *miR-23b* could promote DCs maturation [14]. However, BMSCs with regulatory role for DCs maturation had a high expression of *miR-23b* [15]. Our results showed that the expression of *miR-23b* in BMSCs was significantly higher than that in fibroblasts. In addition, differential expression of *miR-23b* in undifferentiated and differentiated BMSCs was found. So, we speculated that the expression of *miR-23b* was associated with DCs maturation, which was regulated by BMSCs. Further research found that BMSCs had no significant inhibitory effect on the maturation of DCs after *miR-23b* expression was inhibited in BMSCs. Moreover, we obtained the results that the *miR-23b* expression level in BMSCs affected the regulation of DCs on the proliferation of lymphocytes by mixed lymphocyte reaction (MLR). Under the condition of co-culture of BMSCs and DCs, the proliferation of lymphocytes was obviously inhibited, which may be due to the inhibition of DCs maturation; while by down-regulation of miR-23b expression, DCs maturation was not inhibited, and the proliferation of lymphocytes was not significantly inhibited compared with the control group. The experimental results confirmed that BMSCs inhibited the maturation of DCs by overexpression of *miR-23b*.

NF-κB is an effective target for blocking DCs antigen presentation and inhibition dependent on T-cell immune response [29]. The activation of NF-κB is essential for the differentiation and maturation of DCs [30]. Several subunits of NF-κB have been proved to be involved in the functional regulation of DCs [31]. Therefore, we focused on the role of p50 and p65 that were important transcription factors of NF-κB in the mechanism of *miR-23b* regulated DCs maturation. The results showed that in co-culture system as well as the cultured DCs alone, the expression of *miR-23b* was negatively correlated with the expression of p50/p65 both in gene and protein levels. *miR-29a*, *miR-155*, *miR-146a* and *miR-125a-5p* were validated to be significantly differentially expressed in mature DCs compared with iDCs [32]. These studies provided strong evidence that miRNAs were the key regulators in DCs maturation and function. Among them, *miRNA-146a* regulated survival and maturation of DCs via affecting TLR-mediated signalling and TLR-induced NF-κB activation [33]. Moreover, *miR-148/152* can inhibit the production of cytokines including IL-12, IL-6, TNF-α and DC-initiated T-cell proliferation by targeting CaMKIIα [34]. In the present study, *miR-23b* overexpression inhibited the expression of p50/p65, thus blocked the activation of the NF-κB pathway, followed by inhibition of DCs differentiation and maturation.

Through the present study, we confirmed that BMSCs regulated DCs maturation and differentiation through the abnormal expression of *miR-23b*. Further research showed that miR-23b overexpression inhibited the expression of p50/p65, suggesting that the activation of NF-kB was blocked. In conclusion, BMSCs affected the activation of NF-κB pathway through *miR-23b* overexpression and then inhibited the maturation and differentiation of DCs. Our study added new contents to the immune regulation of BMSCs and had important significance for BMSCs application in clinical transplantation therapy.

## Abbreviations

BMSC: bone marrow mesenchymal stem cell
DC: dendritic cell
iDC: immature DC
MSC: mesenchymal stem cell
